# Long non-coding RNA FTH1P3 facilitates uveal melanoma cell growth and invasion through miR-224-5p

This article has been retracted.

**DOI:** 10.1371/journal.pone.0184746

**Published:** 2017-11-02

**Authors:** Xiaoli Zheng, Hongwei Tang, Xiaofeng Zhao, Yamei Sun, Yanfang Jiang, Yonghua Liu

**Affiliations:** 1 Department of Ophthalmology, Liaocheng People's Hospital, Liaocheng, Shandong, China; 2 Joint Laboratory for Translational Medicine, Liaocheng People's Hospital, Liaocheng, Shandong, China; 3 Institute Pasteur of Shanghai Chinese Academy of Science, Shanghai, China; 4 Genetic Diagnosis Center, The First Hospital of Jilin University, Changchun, China; University of South Alabama Mitchell Cancer Institute, UNITED STATES

## Abstract

Growing evidences indicated that Long noncoding RNAs (lncRNAs) played important roles in tumor initiation and progression. However, the function and mechnism of lncRNA ferritin heavy chain 1 pseudogene 3 (FTH1P3) remain unknown in uveal melanoma. We showed that the expression level of FTH1P3 was upregulated in uveal melanoma cell lines and tissues. Elevated expression of FTH1P3 promoted uveal melanoma cell proliferation, cell cycle and migration. Moreover, we found that FTH1P3 was a direct target gene of miR-224-5p in uveal melanoma cell. Overexpression of FTH1P3 suppressed miR-224-5p expression and promoted the expression of Rac1 and Fizzled 5, which were the direct target genes of miR-224-5p. Furthermore, we showed that miR-224-5p expression level was downregulated in uveal melanoma cell lines and tissues. FTH1P3 expression was inversely correlated with the miR-224-5p expression in uveal melanoma tissues. Ectopic expression of miR-224-5p decreased uveal melanoma cell proliferation, cell cycle and migration. Elevated expression of FTH1P3 enhanced uveal melanoma cell proliferation and migration by inhibiting miR-224-5p expression. These results suggest that lncRNA FTH1P3 plays a crucial role in uveal melanoma. Investigation of the underlying mechanism may be a target for the treatment of uveal melanoma.

## Introduction

Uveal melanoma is the most common primary intraocular malignancy cancers with a high mortality of about 50%[1–4]. Early metastasis is the most common cause for the high death rate of this disease[5–7]. Now, no effective treatment is available for patients with metastatic disease because the biology of uveal melanoma initiation and dissemination is unknown[8–10]. Despite several advances in chemotherapy, radiotherapy and surgery, the five year survival rate is still unstatisfied [11–14]. Therefore, it is important to study the molecular event underlying progression and to find the novel therapeutic target of uveal melanoma.

Long noncoding RNAs (lncRNAs) are RNAs with more than 200 nucleotides in length with limited or no protein coding capacity[15–19]. It has been identified that lncRNAs play functional roles in many biological processes such as cell development, proliferation, metastasis, differentiation, invasion and migration[20–24]. Notably, a variety of lncRNAs were found to be deregulated in many tumors such as bladder cancer, glioma, lung cancer, gastric cancer and osteosarcoma[25–29]. FTH1P3 (Ferritin heavy polypeptide 1 pseudogene 3) is one member of the ferritin heavy chain (FHC) gene family[30]. FTH1P3 was found to be upregulated in oral squamous cell carcinoma (OSCC) [31]. Their data suggested that FTH1P3 promoted the OSCC cell progression through inhibiting the miR-224-5p expression and promoting the fizzled 5 expression. However, its function and expression in uveal melanoma are still unknown.

In this study, we tried to study the role of FTH1P3 in uveal melanoma. We found that FTH1P3 expression was overexpressed in uveal melanoma cell lines and tissues. Elevated expression of FTH1P3 increased uveal melanoma cell proliferation, cell cycle and migration.

## Materials and methods

### Tissue samples, cell cultured and transfection

Twenty-five uveal melanoma samples were obtained from uveal melanoma patients and normal uveal tissues were obtained from Beijing Tongren Eye Bank (Beijing, China). All cases provided written informed consent for our study and our study was approved by the Ethics Committee of The Liaocheng People's Hospital. The cell lines (OCM-1A, MUM-2C, C918 and MUM-2B) and melanocyte cell line (D78) were collected from the Chinese Academy of Sciences (Beijing, China) and were cultured in DMEM medium. MiR-224-5p mimic and scramble mimic, pcDNA-FTH1P3 and control vectors were synthesized from Shanghai GenePharma (Shanghai, China). Cell transfection was done using Lipofectamine-2000 (Invitrogen, USA) according to the manufacturer’s protocol. FTH1P3 shRNA: top strand: 5’-CACCGCCAGCCCTCCGTCACCTCTTCGAAAAGAGGTGACGGAGGGCTGGC-3’, and bottom strand: 5’- AAAAGCCAGCCCTCCGTCACCTCTTTTCGAAGAGGTGACGGAGGGCTGGC -3’.

### RNA extraction and qPCR analysis

Total RNA was isolated from cells or samples using the TRIzol reagent kit (Invitrogen, USA) following to manufacturer’s instructions. The expression of FTH1P3, miR-224-5p and Rac1 and fizzled 5 was determined by qRT-PCR with SYBR Green following to the manufacturer’s protocols. The primers were used as following: GAPDH, forward primers 5’-TCACCAGGGCTGCTTTTAAC-3’; reverse primers 5’-GACAAGCTTCCCGTTCTCAG-3’. FTH1P3, forward primers 5’-TCCATTTACCTGTGCGTGGC-3’; reverse primers 5’-GAAGGAAGATTCGGCCACCT-3’. Rac1, forward primers 5’-GGCTAAGGAGATTGGTGCTGTA-3’; reverse primers 5’-ACGAGGGGCTGAGACATTTAC-3’. miR-224-5p forward primer, 5’-CTGGTAGGTAAGTCACTA-3’; reverse primer, 5’-TCAACTGGTGTCGTGGAG-3’.The relative expression of FTH1P3, miR-224-5p and Rac1 and fizzled 5 were measured with the 2^-DDCT^ method. U6 was used as the control for FTH1P3 and miR-224; GAPDH was performed as the control for Rac1 and fizzled 5.

### Cell proliferation, cell cycle and migration

Cell proliferation was determined through using the CCK-8 (Cell Counting Assay Kit-8) (Dojindo, Janpan) following to the manufacturer’s information. Cell proliferation was measured at the time of 0, 24, 48 and 72 hours and the absorbance at 450 nm was analyzed. For cell cycle, the cells fixed in the 70% ethanol and washed in PBS, then re-suspended in the PBS containing RNase, Triton X-100 and propidium iodide (Sigma). The result was analyzed using a Flow Cytometer (BD Biosciences, CA). For cell migration, wound healing assays was performed. The cells were plated in the six-well plate and a wound was created by using the micropipette tip. Photograph was taken immediately and after 48 hours.

### Western blot

Total protein extraction from cells or samples was lysed through using the protein extraction reagent RIPA (Beyotime, China). Equal amounts of protein extractions were resolved by 10% SDS-PAGE and transferred to nitrocellulose membranes (Sigma-Aldrich, USA). After blocking with nonfat milk, membranes were incubated with primary antibodies (fizzled 5, Rac1 and GAPDH, Abcam). Signal was visualized by using ECL (Millipore). GAPDH was performed as the endogenous protein for normalization.

### Statistical analysis

Student’s t-test and one-way ANOVA analysis were used to analyze the data by using the SPSS 18.0 software. Data were shown as mean ±SD. Difference was considered to be statistically significant at p<0.05.

## Results

### FTH1P3 expression level was overexpressed in uveal melanoma cell lines and samples

The expression level of FTH1P3 was upregulated in uveal melanoma cell lines (C918, MUM-2B, OCM-1A and MUM-2C) compared to that in melanocyte cell line (D78) (Fig 1A). In addition, we showed that FTH1P3 expression was higher in uveal melanoma samples than in the non-tumor samples (Fig 1B).

**Fig 1:** FTH1P3 expression level was overexpressed in uveal melanoma cell lines and samples. (A) The FTH1P3 expression in the uveal melanoma cell lines (C918, MUM-2B, OCM-1A and MUM-2C) and melanocyte cell line (D78) was detected by using qRT-PCR. U6 was used as the control. (B) The FTH1P3 expression in the uveal melanoma samples and no-tumor samples was measured by using qRT-PCR. **p<0.01.

### Elevated expression of FTH1P3 increased uveal melanoma cell proliferation and migration

To explore the role of FTH1P3 in uveal melanoma cell, we firstly inforced the FTH1P3 expression in MUM-2B cell using pcDNA-FTH1P3 (Fig 2A). Ectopic expression of FTH1P3 enhanced MUM-2B cell proliferation (Fig 2B). In addition, we found that elevated expression of FTH1P3 promoted the MUM-2B cell cycle (Fig 2C). Moreover, overexpression of FTH1P3 increased the MUM-2B cell migration (Fig 2D). The relative ratio of wound closure per field was shown.

**Fig 2:** Elevated expression of FTH1P3 increased the uveal melanoma cell proliferation and migration. (A) The expression of FTH1P3 in the uveal melanoma cell line MUM-2B treated with pcDNA-FTH1P3 was detected with qRT-PCR. (B) The cell proliferation was meaured by CCK-8 assay. Ectopic expression of FTH1P3 promoted the MUM-2B cell proliferation. (C) Elevated expression of FTH1P3 increased the MUM-2B cell cycle. (D) Wound healing assay was performed to determine the cell migration. (E) The relative ratio of wound closure per field was shown. *p<0.05, **p<0.01 and ***p<0.001.

### FTH1P3 was a direct target gene of miR-224-5p

We used the miRDB (http://mirdb.org/cgi-bin/custom.cgi) to search the target gene of miR-224-5p. As shown in the Fig 3A, FTH1P3 might be a target gene of miR-224-5p. The expression level of miR-224-5p was upregulated in MUM-2B cell after treated with miR-224-5p mimic (Fig 3B). Overexpression of miR-224-5p decreased the luciferase activity of FTH1P3-WT, but not the luciferase activity of FTH1P3-Mut (Fig3C). Elevated expression of miR-224-5p suppressed FTH1P3 expression in MUM-2B cell (Fig 3D).

**Fig 3:** FTH1P3 was a direct target gene of miR-224-5p. (A) MiRDB (http://mirdb.org/cgi-bin/custom.cgi) was used to search the target gene of miR-224-5p. FTH1P3 may be a target gene of miR-224-5p. (B) The expression of miR-224-5p was measured by qRT-PCR. (C) Overexpression of miR-224-5p decreased the luciferase activity of FTH1P3-WT, but it has not decreased the luciferase activity of FTH1P3-Mut. (D) Overexpression of miR-224-5p decreased the FTH1P3 expression in the MUM-2B cell.

### Overexpression of FTH1P3 decreased miR-224-5p expression

Elevated expression of FTH1P3 suppressed miR-224-5p expression in the MUM-2B cell (Fig 4A). FTH1P3 overexpression enhanced Rac1 expression in the MUM-2B cell (Fig 4B). Ectopic expression of FTH1P3 promoted Fizzled 5 expression (Fig 4C). The protein expression of Rac1 (Fig 4C) and Fizzled 5 (Fig 4D) was also upregulated.

**Fig 4:** Overexpression of FTH1P3 decreased the miR-224-5p expression. (A) Elevated expression of FTH1P3 decreased the miR-224-5p expression in the MUM-2B cell. (B) FTH1P3 overexpression promoted the expression of Rac1. (C) Overexpression of FTH1P3 enhanced the Fizzled 5 expression. (D) The protein expression of Rac1 was measured by western blot. FTH1P3 overexpression promoted the protein expression of Rac1. (E) The protein expression of Fizzled 5 was measured by western blot.

### MiR-224-5p expression level was downregulated in uveal melanoma cell lines and samples and inversely correlated with FTH1P3

The expression level of miR-224-5p was downregulated in uveal melanoma cell lines (C918, MUM-2B, OCM-1A and MUM-2C) compared to the melanocyte cell line (D78) (Fig 5A). In addition, we showed that miR-224-5p expression was lower in uveal melanoma samples than in the non-tumor samples (Fig 5B). In addition, the expression of miR-224-5p in uveal melanoma tissues was inversely correlated with FTH1P3 expression (Fig 5C).

**Fig 5:** miR-224-5p expression level was downregulated in uveal melanoma cell lines and samples and inversely correlated with FTH1P3. (A) The expression level of miR-224-5p in the uveal melanoma cell lines (C918, MUM-2B, OCM-1A and MUM-2C) and melanocyte cell line (D78) was determined by qRT-PCR. (B) The miR-224-5p expression was lower in the uveal melanoma samples than in the no-tumor samples. (C) The expression of miR-224-5p in the uveal melanoma tissues was inversely correlated with FTH1P3 expression. ***p<0.001.

### FTH1P3 enhanced uveal melanoma cell proliferation and migration by inhibiting the miR-224-5p expression

Ectopic expression of miR-224-5p suppressed MUM-2B cell proliferation (Fig 6A). Moreover, elevated expression of miR-224-5p inhibited MUM-2B cell cycle (Fig 6B). MiR-224-5p overexpression decreased MUM-2B cell migration and the relative ratio of wound closure per field was shown (Fig 6C). Next, we restored miR-224-5p expression through transfecting with miR-224-5p mimic into the FTH1P3 overexpressing-MUM-2B cells. The advantageous role of FTH1P3 on the MUM-2B cell proliferation was reversed by miR-224-5p overexpression (Fig 6D). Overexpression of miR-224-5p decreased the cell cycle in the FTH1P3 overexpressing-MUM-2B cell (Fig 6E). Ectopic expression of miR-224-5p suppressed the cell migration in the FTH1P3 overexpressing-MUM-2B cell (Fig 6F).

**Fig 6:** FTH1P3 enhanced the uveal melanoma cell proliferation and migration by inhibiting the miR-224-5p expression. (A) Ectopic expression of miR-224-5p suppressed the MUM-2B cell proliferation. (B) Overexpression of miR-224-5p suppressed the MUM-2B cell cycle. (C) Ectopic expression of miR-224-5p decreased the MUM-2B cell migration and the relative ratio of wound closure per field was shown in the right. (D) We restored miR-224-5p expression through transfecting miR-224-5p mimic into the FTH1P3 overexpressing-MUM-2B cells. The advantageous role of FTH1P3 on the MUM-2B cell proliferation was reversed by miR-224-5p overexpression. (E) Overexpression of miR-224-5p decreased the cell cycle in the FTH1P3 overexpressing-MUM-2B cell. (F) Ectopic expression of miR-224-5p suppressed the cell migration in the FTH1P3 overexpressing-MUM-2B cell. The relative ratio of wound closure per field was shown in the right. *p<0.05, **p<0.01 and ***p<0.001.

## Discussion

Increasing evidences showed lncRNAs played important roles in many tumor cellular processes such cell cycle, proliferation, survival, invasion and migration[32–37]. Until now, the mechanism and effect of lncRNAs are largely unclear in uveal melanoma tumorigenesis and progression. LncRNA FTH1P3 is one member of lncRNAs located in the 2p23.3 with a length of 954 nucleotides[38]. Previous studies suggested that FTH1P3 acted as an oncogene in oral squamous cell carcinoma[31]. Zhang et al[31]. showed that FTH1P3 expression level was highly expressed in oral squamous cell carcinoma.Di et al[38]. reported that FTH1P3 transcript was found in many tissues and cell lines and the expression of FTH1P3 was positively regulated during cell differentiation process. In addition, Zhang et al[30]. demonstrated that FTH1P3 was upregulated in oral squamous cell carcinoma tissues. Overexpression of FTH1P3 enhanced oral squamous cell carcinoma cell colony formation and proliferation by regulating the expression of miR-224-5p and Fizzled 5. To our knowledge, there are no references about the role of FTH1P3 in uveal melanoma.

In the current study, we showed that FTH1P3 expression was overexpressed in uveal melanoma cell lines and tissues. Elevated expression of FTH1P3 increased uveal melanoma cell proliferation, cell cycle and migration. Moreover, we found that FTH1P3 was a direct target gene of miR-224-5p in uveal melanoma cell. Overexpression of FTH1P3 decreased miR-224-5p expression and promoted the expression of Rac1 and Fizzled 5, which were the direct target genes of miR-224-5p. Furthermore, we showed that miR-224-5p expression level was downregulated in uveal melanoma cell lines and tissues. The expression level of miR-224-5p was inversely correlated with FTH1P3 in uveal melanoma tissues. Ectopic expression of miR-224-5p decreased uveal melanoma cell proliferation, cell cycle and migration. Elevated expression of FTH1P3 enhanced the uveal melanoma cell proliferation and migration by inhibiting miR-224-5p expression.

Previous studies suggested that lncRNAs acted as sponges for miRNAs and abolished the suppressive effect of miRNAs on the targeted transcripts[39, 40]. Previous study showed that FTH1P3 overexpression promoted oral squamous cell carcinoma progression through acting as a molecular sponge of miR-224-5p[31]. In line with this, we also showed that elevated expression of FTH1P3 suppressed the miR-224-5p expression in uveal melanoma cell. Moreover, we demonstrated that FTH1P3 overexpression promoted the expression of Rac1 and Fizzled 5, which were the target genes of miR-224-5p. Previous studies suggested that miR-224 played important roles in the tumor initiation and progression[41–43]. For example, Wang et al[44]. demonstrated that miR-224-3p expression was upregulated in HPV-infected tissues and cell lines. Overexpression of miR-224-3p inhibited the hrHPV-induced cervical cancer cell autophagy by targeting FAK family-interacting protein of 200 kDa (FIP200). Liu et al[45]. showed that miR-224 suppressed breast cancer cell migration and proliferation by inhibiting Fizzled 5 expression. Geng et al[46]. showed that miR-224 expression was decreased in osteosarcoma tissues and cell lines. Overexpression of miR-224 inhibited osteosarcoma cell migration, proliferation and invasion and contributed to the enhanced sensitivity of the osteosarcoma cells to cisplatin by regulating Rac1 expression. However, the function and mechanism of miR-224 in the uveal melanoma remain unknown. In this study, we demonstrated that the miR-224-5p expression level was downregulated in uveal melanoma cell lines and tissues. Interestingly, we showed that the expression of miR-224-5p was inversely correlated with FTH1P3 in uveal melanoma tissues. Moreover, ectopic expression of miR-224-5p suppressed uveal melanoma cell proliferation, cell cycle and migration. In addition, ectoptic expression of FTH1P3 promoted uveal melanoma cell proliferation, cell cycle and migration through inhibiting miR-224-5p expression.

In conclusion, we demonstrated that lncRNA FTH1P3 was commonly up-regulated in uveal melanoma cell lines and tissues and acted as an oncogene in uveal melanoma progression by inhibiting miR-224-5p expression. These results suggest that lncRNA FTH1P3 plays a crucial role in uveal melanoma and investigation of the underlying mechanism may be a target for the treatment of uveal melanoma.
